The article "Application of Data Mining Algorithms for Dementia in People with HIV/AIDS" was published in 2021. Journal: Comput Math Methods Med.

# Application of Data Mining Algorithms for Dementia in People with HIV/AIDS

**DOI:** 10.1155/2021/4602465

**Published:** 2021-07-09

**Authors:** Luana Ibiapina Cordeiro Calíope Pinheiro, Maria Lúcia Duarte Pereira, Marcial Porto Fernandez, Francisco Mardônio Vieira Filho, Wilson Jorge Correia Pinto de Abreu, Pedro Gabriel Calíope Dantas Pinheiro

**Affiliations:** ^1^Graduate Program in Clinical Care in Nursing and Health, State University of Ceará, Fortaleza, Brazil; ^2^Graduate Program in Computer Science, State University of Ceará, Fortaleza, Brazil; ^3^Porto School of Nursing, Porto, Portugal; ^4^Graduate Program in Applied Informatics, University of Fortaleza, Fortaleza, Brazil

## Abstract

Dementia interferes with the individual's motor, behavioural, and intellectual functions, causing him to be unable to perform instrumental activities of daily living. This study is aimed at identifying the best performing algorithm and the most relevant characteristics to categorise individuals with HIV/AIDS at high risk of dementia from the application of data mining. Principal component analysis (PCA) algorithm was used and tested comparatively between the following machine learning algorithms: logistic regression, decision tree, neural network, KNN, and random forest. The database used for this study was built from the data collection of 270 individuals infected with HIV/AIDS and followed up at the outpatient clinic of a reference hospital for infectious and parasitic diseases in the State of Ceará, Brazil, from January to April 2019. Also, the performance of the algorithms was analysed for the 104 characteristics available in the database; then, with the reduction of dimensionality, there was an improvement in the quality of the machine learning algorithms and identified that during the tests, even losing about 30% of the variation. Besides, when considering only 23 characteristics, the precision of the algorithms was 86% in random forest, 56% logistic regression, 68% decision tree, 60% KNN, and 59% neural network. The random forest algorithm proved to be more effective than the others, obtaining 84% precision and 86% accuracy.

## 1. Introduction

Data mining (MD) is one of the data exploration processes capable of predicting and extracting consistent patterns by using strategies such as learning algorithms, such as artificial intelligence (AI), or classification in statistics, which can reveal hidden relationships and accurate data [1, 2].

The application of MD is in health information systems, in the public and private spheres, which, through a process of selection, preprocessing, and data transformation, one can discover patterns and generate knowledge through their interpretations. With this method, the health professional will identify, characterise, and guide the patient based on patterns of health problems and care therapies for different diseases [2].

The article "Application of Data Mining Algorithms for Dementia in People with HIV/AIDS" was published in 2021. Journal: Comput Math Methods Med.

As one of the most prevalent diseases and considered a public health problem, we have neurocognitive disorders associated with the human immunodeficiency virus (HAND) because of the virus compromising the immune system. Also, it has an affinity for the central nervous system (CNS) by destroying macrophages that cross the blood-brain barrier, which cannot be invaded by highly active antiretroviral therapy (HAART) [3, 4].

Among the cognitive disorders associated with the human immunodeficiency virus (HIV), dementia is considered its most serious type, as it interferes with the motor, behavioural, and intellectual functions of the infected individual, causing him the inability to perform instrumental activities of daily living, whose symptoms are manifested by irritability, emotional lability, memory loss, dysdiadochokinesia, and spastic gait [5, 6].

The health professional, despite carrying out the clinical history, neurological, and cognitive examination, sometimes feels undecided as to the therapeutic approach to be taken in the face of a possible neurological complication, since the onset of HIV dementia is insidious and initial symptoms may be confused with other psychiatric illnesses, such as depression and anxiety [7].

In this context, the use of technological strategies, such as information and communication technologies (ICT), can be considered essential tools for detecting the early diagnosis of dementia and other diseases. Computer science methodologies with ICT may be able to classify the main characteristics of the disease, in the face of the patient's social and clinical changes, in a practical way and serve as an aid for health professionals in promoting information management and quality safe care [8].

Among the computational techniques, there is the use of algorithms that consists of the understanding and structure of existing data and capable of generating predictive rules, whose results, when combined, can bring benefits in reducing costs and in the effectiveness of interventions, both in treatment and in preventive actions [9].

Thus, the following question arises: can a data mining technique identify the most relevant characteristics given the risk of dementia in people with HIV/AIDS?

Early recognition and categorisation of the characteristics that influence the risk of dementia will allow the ability to reverse the disease to choose an effective HAART and additional treatments through better social and psychological support to improve the person's life expectancy and quality life with HIV/AIDS. It will also assist the health professional by offering more precise and targeted guidance to family members in the face of behavioural and cognitive changes of the seropositive individual.

The article "Application of Data Mining Algorithms for Dementia in People with HIV/AIDS" was published in 2021. Journal: Comput Math Methods Med.

For some years, predictive models have been developed to predict outcomes of interest to the population's health, like computerised image analysis based on precision medicine. Researchers believed that the machine could interpret the analysis of complex and straightforward testing [10].

Besides, contributing to the agility in the interpretation of results by reducing the time of action for urgent cases and increasing the degree of confidence in the diagnoses is an advantage of the technologies applied to health, together with the presence of the health professional during the verification and validation of the results based on clinical, epidemiological correlations, and therapeutic decision [10].

In this context, more flexible artificial intelligence algorithms have been used in predictive modelling of outcomes of health interest due to the high amount of data available to carry out this research. As a result, the algorithms show a better outcome prediction potential because they capture complex relationships in the data and their ability to deal with many predictors [11, 12].

Regarding sexually transmitted infections to affected people, prognostic information related to the risk of death and other opportunistic diseases has become increasingly important for health professionals. Also, researchers and public policymakers are a tool to assist in decision-making regarding disease tracking targeting preventive programs and offering specialised treatments [10].

In this context, the study seeks to identify the algorithm with the best performance capable of revealing the most relevant characteristics in the high risk of developing dementia in people with HIV/AIDS, based on data mining.

## 2. Methodology

In this research, the principal component analysis (PCA) algorithm was applied to assess the impact of reduced dimensionality and the quality of the solution between the following machine learning algorithms: logistic regression, decision tree, neural network, KNN, and forest random.

Machine learning algorithms have specific functions, such as logistic regression, whose statistical technique describes the behaviour between a binary dependent variable and independent metric or nonmetric variables. It investigates the effect of the variables by which individuals are exposed to the probability of a specific event occurring [10].

The decision tree is a nonparametric method applied for data classification and regression, in which a set of attributes is used to predict an output value. The model is formed by elements with information called nodes, which are read in a descending way, and which starts at the root node, with a higher hierarchical level until it reaches the leaf node that consists of the output, that is, the predicted result [10–12].

The article "Application of Data Mining Algorithms for Dementia in People with HIV/AIDS" was published in 2021. Journal: Comput Math Methods Med.

Neural network seeks to simulate the processes of a human neural network through models composed of nonlinear elements that operate in parallel, through the environment and ends when the neural network manages to generalise solutions for a class of problem [13].

The KNN algorithm is a learning based on instances stored. As a new sample is presented to the algorithm, a new classification is generated from a distance closest to neighbouring cases. The decision rule is built directly without estimating the densities conditioned to the classes; relative patterns can be classified in the space of characteristics that probably belong to the same class [13–15].

The random forest consists of a set of decision trees generated within the same object, using a classifier aggregation technique built so that its structure is composed at random. Thus, the method combines several decision trees through a vote that classifies the final class to receive the highest votes [2].

The database used for this study was built by collecting data from 270 HIV/AIDS-infected individuals and followed up at the outpatient clinic of a Reference Hospital for Infectious and Parasitic Diseases, in the State of Ceará, Brazil, from January to April 2019. The questionnaire used for the collection was composed of sociodemographic data, clinical health, and risk behaviours; simplified medication adherence questionnaire (SMAQ), Brazilian version to assess adherence to treatment with antiretrovirals; the International Dementia Scale to detect dementia in the HIV patient; the Barthel Index and the Lawton and Brody Scale to assess the degree of functional capacity; and finally the Social Support Scale for people living with HIV/AIDS.

The International HIV-Associated Dementia Scale (IHDS) is a screening tool to identify the high or low risk of dementia in HIV patients who do not need a specialist and are not influenced by the individual's education. Also, the use of the scale in clinical practice has a sensitivity of approximately 80% and specificity around 57%, with a cut-off score less than or equal to 10 for HAD diagnosis. IHDS can be used to identify probable cases of HAD in situations where formal neuropsychological assessment is impossible.

Table 1 shows the classes with the most relevant independent variables used in this research:

The Python programming language is versatile and capable of providing good code performance and readability. This language is viable for working with rapid application development methods, reducing waste, and optimising code quality; development techniques “are not repeated” and do not allow ambiguities, and have fast and straightforward software [15].

The article "Application of Data Mining Algorithms for Dementia in People with HIV/AIDS" was published in 2021. Journal: Comput Math Methods Med.

The study was carried out from the execution of all the machine learning algorithms already mentioned. It sought to analyse the performance of the algorithms from the 104 available characteristics present in the database.

Before executing the PCA, the data were standardised using the mean and standard deviation, according to the following equation:

(1) $$\begin{array}{c} z=\frac{x–\mu }{\sigma }, \end{array}$$

where *μ* is the mean and *σ* is the standard deviation applied in the execution of machine learning algorithms.

Subsequently, the principal component analysis (PCA) algorithm was performed, whose multivariate statistical technique is widely used to reduce dimensions and extract resources. The processing of this technique can be summarised as a set of orthogonal linear transformations of the original variables so that the transforming variables maintain, as much as possible, the information contained in the actual characteristics [1, 16].

The PCA captured 90% of the variation in the data and selected the main characteristic of each of these components without repetition.

In the third moment, the main components were analysed, which captured 80% of the data variation and selected the main characteristic of each one without repetition.

They sorted the components in descending order by the variation of the data they represented. Thus, the first components reflected the most significant relevance and corresponded to most of the data variation.

For each of these executions, we analysed the performance of the algorithms and the respective most representative characteristics.

## 3. Results and Discussion

Initially, the logistic regression, decision tree, neural network, KNN, and random forest algorithms were obtained for 104 components, with the following results in Table 2.

The total execution time of the algorithms took a maximum of 03 seconds, which corresponded from reading and processing the database to reading the PCA. It should be noted that each algorithm independently took up to 02 seconds to obtain the results.

Through the PCA, the number of characteristics was reduced from 104 to 47. Generally, there was a reduction in the performance of the algorithms; random forest, for example, started to reach 80.49% accuracy, and therefore, the number of characteristics was reduced from 47 to 33.

The article "Application of Data Mining Algorithms for Dementia in People with HIV/AIDS" was published in 2021. Journal: Comput Math Methods Med.

Moreover, the performance of the algorithms remained as in the execution already mentioned, except Logistic regression continued to lose performance.

Logistic regression continued to lose performance. The following steps were performed considering the main components that captured 70%, 60%, 50%, and 40% of data variation, respectively, when observed in Table 3.

Figure 1 shows that 70% captured from 23 characteristics were analysed; the accuracy of the different algorithms showed the best performance of random forest:

From the results obtained in the executions carried out, it is possible to analyse approximately 86% in random forest, 56% logistic regression, 68% decision tree, 60% KNN, and 59% neural network.

Dimensionality reduction could improve the quality of machine learning algorithms. It delimits the less relevant components that will only cause noise in the algorithms or increase the complexity of the problem. However, ignoring elements causes some of the data variation to be lost, leading to reduced performance of the prediction algorithms.

It can be seen in Figure 2 that during the tests, even losing about 30% of the data variation, that is, when considering only 23 characteristics, the random forest algorithm obtained better results regarding the precision and accuracy of 84% and 86%, respectively. In different areas of study, random forest has obtained good results and demonstrated that these algorithms had provided superior results in the prediction capacity compared to other machine learning algorithms. Moreover, it can analyse from samples considered small like this one study until analysing complex data structures [17, 18].

It is also noted that when using less than 23 characteristics, the algorithm loses performance, which assumes that essential aspects may be being disregarded. Reducing the dimensionality of PCA has reduced the complexity of the data and filters out the crucial characteristics to classify whether a patient is at risk of developing dementia.

Thus, the main characteristics extracted with this technique are described below, in an increasing order of representativeness of the data: paranoid ideation; walking; adherence to antiretroviral medication; having the impression that something is wrong in your head or your spirit; having terror or panic attacks; TCD4+lymphocyte values at the first consultation; HIV infection time; type of vírus; previous hospitalisation due to HIV infection; anxiety; coinfection with the hepatitis B vírus; does not use antiretroviral medication; feeling of sadness and loneliness; interruption of drug treatment; Barthel category; age; use of antiretroviral medication; viral load at the first visit; hopeless about the future; the presence of opportunistic diseases; having the idea that other people are to blame for most of their problems; bladder control; and schooling.

The article "Application of Data Mining Algorithms for Dementia in People with HIV/AIDS" was published in 2021. Journal: Comput Math Methods Med.

Psychopathological symptoms can be assessed by the Brief Symptom Inventory indicator, whose nine dimensions are elements of psychopathology, such as somatisation that reveals complaints from cardiovascular to gastrointestinal; obsession-compulsion, obsession-compulsion is a symptom of the individual's impulsive behaviour. Interpersonal sensitivity, which turns to the feeling of inferiority and shyness; depression; anxiety, which can be assessed through nervous manifestations and apprehension; hostility; phobic anxiety; paranoid ideation, whose behaviour is considered harmful and disturbing; and psychoticism, in which the individual isolates himself and has schizophrenic behaviours, through hallucinations [19, 20].

Phobic conditions such as terror or panic attacks may require the individual to overestimate the danger offered by the object or event in question since the discovery of HIV infection, as well as the infection's relationship with certain mental illnesses, given the neuroinflammatory factors and the stress that contribute to this situation [19–21].

Depression is one of the most common comorbidities in HIV-positive patients, causing worsening of medication adherence and increased mortality. Clinical findings demonstrate a relationship between depression and increased levels of inflammatory cytokines (TNF-alpha, IL-1beta, and IL-6) in both systemic and CSF terms [19–21].

Among the feelings of sadness and loneliness related to a depressive condition, it can be associated with factors other than disease progression. The depressive feeling persists when the subject reveals a lack of hope for the future, thereby affecting adherence to antiretrovirals [21].

The low antiretroviral adhesion directly implies the cognitive damages caused by the high viral load and the degree of immunosuppression of the infected individual, whose determinant most susceptible to HAND corresponds to the nadir values of LTCD4 + <350 cells/mm^3^ or LTCD4 + current < 350 cells/mm^3^ [22, 23].

Also, it is emphasised about opportunistic neurological diseases of HIV, such as neurotoxoplasmosis, tuberculous meningitis, and neurocryptococcosis, which are essential comorbidities for psychiatric damage. Neurotoxoplasmosis is the most frequent opportunistic infection in the CNS in HIV-positive individuals, causing a lesion with a more common mass effect, especially when the patient has CD4 + <200 cells/mm^3^ [22–26].  Table 4 presents the demographic characteristics of people with HIV according to the research covered.

The article "Application of Data Mining Algorithms for Dementia in People with HIV/AIDS" was published in 2021. Journal: Comput Math Methods Med.

The predominant sociodemographic characteristics in this research were people with HIV (male) (66.29%), aged between 50 and 55 years old (49.25%), single (53.33%), and with a low level of education (33%).

Regarding age, scientific evidence reveals that the proportion of older adults living with HIV in the Netherlands in 2030 will reach 73%. In the United States of America (USA) and Brazil, it currently exceeds 50%. Among the statistics, half of HIV infections in older women are acquired at approximately 56 years. Thus, age can be considered significant when associated with HIV, given the high probability of late diagnosis and short-term mortality [27].

In terms of schooling, theoretical studies investigate the relationship between the level of knowledge and its influence on health behaviour in the awareness of self-perceived risk, continued condom use during sexual intercourse, and adherence to antiretroviral drug therapy [28].

Thus, people with a low level of education need social support and continuous monitoring by health professionals regarding the assessment of precession, which is permanently monitored in the evaluation of the information they understand and its impact on the quality of life in the dimensions: social, cultural, psychic, and clinical [28].

In this way, the practical and early diagnosis of these neuropsychological conditions and the correct therapeutic intervention can delay or even reverse dementia associated with HIV and benefit the individual.

## 4. Conclusion and Future Works

Because of the database used, it was possible to classify and analyse the main characteristics of dementia in people with HIV/AIDS using techniques such as PCA and MD. Through computational tests between the MD algorithms, the random forest algorithm proved to be more effective concerning the others, obtaining higher precision and accuracy.

In addition to dementia, this research could be insightful about other mental disorders in the face of initial symptoms of depression, panic attacks, and feelings of persecution. Thus, it may be able to sensitise health professionals to a more accurate assessment of factors related to the individual's personality, which may be associated with medication adherence and, consequently, with the value of viral load and TCD4 lymphocytes.

Thus, identifying the main characteristics of prediction of dementia due to HIV can assist the health professional for referral and appropriate treatment to these infected people through interpersonal, cognitive-behavioural, and supportive psychotherapy. In addition, orientation contributing to the family about adherence to antiretroviral therapy monitoring, social life, and instrumental activities by the HIV-positive individual.

The article "Application of Data Mining Algorithms for Dementia in People with HIV/AIDS" was published in 2021. Journal: Comput Math Methods Med.

Since the results of this application are in a local population, it is suggested that these algorithms be applied to more massive databases to confirm and improve their performance. Although the sample is small, its data is independent and distributed equally about those observed in the future and follow the same distribution of the population from which the sample was taken.

## Figures and Tables

**Figure 1:** Accuracy of machine learning algorithms regarding HIV-associated dementia characteristics.

**Figure 2:** Precision ratio, accuracy, and recall of random forest using different amounts of features.

**Table 1:** Classes and independent variables of people with HIV/AIDS.

Classes	Variables
Sociodemographic profile	Age, gender, marital status, education

History of infectious disease	Transmission route, virus type, years with HIV, hepatitis B, hepatitis C, comorbidities, previous hospitalisation, opportunistic disease, initial viral load, current viral load, initial TCD4, current TCD4

Drug adherence	Antiretroviral, forgets to use medication, careless use of medication, stops drug therapy

Neurological assessment	Heads up, psychomotor speed, memory, construction

Psychosomatic changes	Anxiety, obsession-compulsion, interpersonal sensitivity, depression, summing, psychoticism, phobic anxiety, hostility, paranoid ideation

Daily activities	Food, wear, bath, hygiene, going to the bathroom, intestinal control, bladder control, climbing ladder, get up, wander

**Table 2:** Analysis of machine learning algorithms against the variation of HIV-associated dementia data.

Total features: 104	Logistic regression	Decision tree	Neural network	KNN	Random forest
No PCA					
Accuracy	0.7805	0.7317	0.5732	0.6098	0.8293
Precision	0.7377	0.7451	0.5732	0.6415	0.7797
Recall	0.9574	0.8085	1.0	0.7234	0.9787

**Table 3:** Analysis of machine learning algorithms against the variation of HIV-associated dementia data.

		Logistic regression	Decision tree	Neural network	KNN	Random forest
Total features: 104						
No PCA	Accuracy	0.7805	0.7317	0.5732	0.6098	0.8293
	Precision	0.7377	0.7451	0.5732	0.6415	0.7797
	Recall	0.9574	0.8085	1.0	0.7234	0.9787

Total features: 47 (PCA = 90%)						
90% of captured variation	Accuracy	0.7439	0.7073	0.5732	0.5976	0.8049
	Precision	0.7097	0.7091	0.5732	0.6296	0.7627
	Recall	0.9362	0.8298	1.0	0.7234	0.9574

Total features: 33						
80% of captured variation	Accuracy	0.7195	0.7683	0.5610	0.5976	0.8049
	Precision	0.6935	0.7917	0.7619	0.6296	0.7541
	Recall	0.9149	0.8085	0.3404	0.7234	0.9787

Total features: 23						
70% of captured variation	Accuracy	0.5610	0.6829	0.5854	0.5976	0.8659
	Precision	0.5679	0.6981	0.9333	0.6296	0.8462
	Recall	0.9787	0.7872	0.2979	0.7234	0.9362

Total features: 16						
60% of captured variation	Accuracy	0.7317	0.7073	0.6463	0.5366	0.8049
	Precision	0.7049	0.7447	0.7500	0.5957	0.7818
	Recall	0.9149	0.7447	0.5745	0.5957	0.9149

Total features: 10						
50% of captured variation	Accuracy	0.7195	0.6098	0.5610	0.5122	0.7317
	Precision	0.7000	0.6667	0.5696	0.5714	0.7358
	Recall	0.8936	0.6383	0.9574	0.5957	0.8298

Total features: 6						
40% of captured variation	Accuracy	0.6220	0.5610	0.5366	0.5000	0.6829
	Precision	0.6111	0.6279	0.5570	0.5600	0.7059
	Recall	0.9362	0.5745	0.9362	0.5957	0.7660

The article "Application of Data Mining Algorithms for Dementia in People with HIV/AIDS" was published in 2021. Journal: Comput Math Methods Med.

**Table 4:** Demographic characteristics of people with HIV.

Gender	Female	91
	Male	179

Age	50 to 55	133
	56 to 60	75
	61 to 70	52
	>70	10

Marital status	Not married	114
	Married	71
	Widowed	43
	Divorced	42
	Incomplete fundamental	89

Education	Completed elementary school	46
	High school	61
	Higher	29
	Illiterate	45

## Data Availability

The data [database] used to support the conclusions of this study are available from the corresponding author upon request.

## References

[1] Blazhenets G., Ma Y., Sörensen A. (2019). Principal components analysis of brain metabolism predicts development of Alzheimer dementia. *Journal of Nuclear Medicine*.

[2] Tabib S., Larocque D. (2020). Non-parametric individual treatment effect estimation for survival data with random forests. *Bioinformatics*.

[3] Graciela P. S. (2019). Trastornos neurocognitivos en pacientes con VIH datos preliminares de uma cohorte prospectiva uruguaya. *Revista Medica Del Uruguay*.

[4] Airoldi M., Bandera A., Trabattoni D. (2012). Neurocognitive impairment in HIV-infected naïve patients with advanced disease: the role of virus and intrathecal immune activation. *Clinical & Developmental Immunology*.

[5] Perdigão R. E. A., Bonolo P. d. F., Silveira M. R., Silva D. I. d., Ceccato M. d. G. B. (2020). Oportunidade de vinculação de pessoas vivendo com HIV em um serviço especializado de saúde, Belo Horizonte (MG). *Revista Brasileira de Epidemiologia*.

[6] Saylor D., Dickens A. M., Sacktor N. (2016). HIV-associated neurocognitive disorder -- pathogenesis and prospects for treatment. *Nature Reviews Neurology*.

[7] Deus D. M. V., Possas C. C. (2018). Atualizações sobre demência cortical em indivíduos infectados pelo HIV. *Humanae*.

[8] Silveira F. R. V., Moreira L. Y. M. R. (2020). Use of machine learning algorithms in the prediction of Aedes aegypti transmitted arboviruses. *Conexoes - Ciencia e Tecnologia*.

[9] Tamanini I., Pinheiro P. R., dos Santos C. N. (2012). A hybrid approach of verbal decision analysis and machine learning. *Lecture Notes in Computer Science*.

The article "Application of Data Mining Algorithms for Dementia in People with HIV/AIDS" was published in 2021. Journal: Comput Math Methods Med.

[10] Santos K. M., Ferreira Júnior J. R., Wada D. T., Tenório A. P. M., Barbosa M. H. N., Marques P. M. d. A. (2019). Artificial intelligence, machine learning, computer-aided diagnosis, and radiomics: advances in imaging towards to precision medicine. *Radiologia Brasileira*.

[11] Obermeyer Z., Emanuel E. J. (2016). Predicting the future: big data, machine learning, and clinical medicine. *The New England Journal of Medicine*.

[12] Maia C. M., Gomes J. C. M., Chagas L. D. (2017). Estudo sobre o uso de árvores de decisão na área da saúde. *Anais do Encontro de Computação do Oeste Potiguar ECOP/UFERSA*.

[13] Jamei M., Nisnevich A., Wetchler E., Sudat S., Liu E. (2017). Predicting all-cause risk of 30-day hospital readmission using artificial neural networks. *PLoS One*.

[14] Olivera A. R., Roesler V., Iochpe C. (2017). Comparison of machine-learning algorithms to build a predictive model for detecting undiagnosed diabetes - ELSA-Brasil: accuracy study. *Sao Paulo Medical Journal*.

[15] Silva I. R. S., Silva R. O. (2019). Python programming language. *Revista Tecnologias em Projeção*.

[16] Faria M. M. (2016). *Detecção de intrusões em redes de computadores com base nos algoritmos KNN, K-Means++ e J48*.

[17] Géron A. (2017). *Hands-On Machine Learning with Scikit-Learn and Tensor Flow: Concepts, Tools, and Techniques to Build Intelligent Systems*.

[18] Raschka S., Mirjalili V. (2017). *Python Machine Learning*.

[19] Derogatis L. (1982). *The Brief Symptom Inventory (BSI): Administration and Procedures–Manual*.

[20] Sanabria-Mazo J. P., Hoyos-Hernández P. A., Bravo F. (2020). Psychosocial factors associated with HIV testing in Colombian university students. *Acta Colombiana de Psicología*.

[21] Ayele B. A., Amongne W., Gemechu L. (2020). HIV-associated neurocognitive disorder and HIV-associated myelopathy in a patient with a preserved CD4, but high viral load-a rarely reported phenomenon: a case report and literature review. *BMC Infectious Diseases*.

[22] Heaton R. K., Franklin D. R., Deutsch R. (2015). Neurocognitive change in the era of HIV combination antiretroviral therapy: the longitudinal charter study. *Clinical Infectious Diseases*.

[23] Serrano-Villar A. R. S., Gutierrez F., Mirall E. S. C. (2016). HIV as a chronic disease: evaluating and managing non-AIDS defining. *Management of HIV-Associated Disease in HIV*.

[24] Sacktor N. (2018). Changing clinical phenotypes of HIV-associated neurocognitive disorders. *Journal of Neurovirology*.

[25] Camargo L. A., Capitão C. G., Filipe E. M. V. (2014). Saúde mental, suporte familiar e adesão ao tratamento: associações no contexto HIV/AIDS. *Psico-USF*.

[26] Ouyang Y., Liu L., Zhang Y. (2014). Discordant patterns of tissue-specific genetic characteristics in the HIV-1 env gene from HIV-associated neurocognitive disorder (HAND) and non-HAND patients. *Journal of Neurovirology*.

The article "Application of Data Mining Algorithms for Dementia in People with HIV/AIDS" was published in 2021. Journal: Comput Math Methods Med.

[27] Cruz G. E. C. P., Cardoso D. F. B., da Silva E. S., Silveira R. C. P., Silva A. E., Apostolo J. L. A. (2020). Late diagnosis of human immunodeficiency virus and acquired immunodeficiency syndrome in the elderly: scoping review protocol. *Enfermería Actual de Costa Rica*.

[28] de Freitas Magalhães Gomes R. R., das Graças Braga Ceccato M., Kerr L. R. F. S., Guimarães M. D. C. (2017). Factors associated with low knowledge on HIV/AIDS among men who have sex with men in Brazil. *Cadernos de Saúde Pública*.

